The article "MicroRNA‐498 reduces the proliferation and invasion of colorectal cancer cells via targeting Bcl‐2" was retracted in 2024. Reasons: duplicated images; unreliable data; unreliable results or conclusions.

# MicroRNA‐498 reduces the proliferation and invasion of colorectal cancer cells via targeting Bcl‐2

**DOI:** 10.1002/2211-5463.12767

**Published:** 2019-12-17

**Authors:** Tongsheng Wang, Ling Ma, Wenxia Li, Lei Ding, Hong Gao

**Affiliations:** ^1^ Department of Colorectal Tumor Surgery Beijing Shijitan Hospital Affiliated to Capital Medical University China

**Keywords:** apoptosis, Bcl‐2, colorectal cancer, miR‐498

## Abstract

Colorectal cancer (CRC) remains a major cause of carcinoma‐related deaths worldwide. MicroRNA‐498 (miR‐498) modulates the development of a variety of biological events, including tumorigenesis. Nevertheless, it is unclear whether miR‐498 plays a role in CRC. This study was designed to elucidate the underlying mechanism and role of miR‐498 in modulation of the viability and invasiveness of CRC cells. We report that CRC tissues and cells exhibited decreased expression of miR‐498, and that overexpression of miR‐498 resulted in reduced proliferation of CRC cells, concomitant with increased apoptosis. Furthermore, bioinformatic prediction and dual‐luciferase reporter assay revealed that miR‐498 targeted the 3′‐UTR of Bcl‐2 for silencing. However, Bcl‐2 overexpression suppressed the proapoptosis of miR‐498 on CRC cells. In summary, we describe a possible role of miR‐498 in CRC, which may lead to the identification of new targets for treatment of this malignancy.

## Graphical abstract

In colorectal cancer cells, miR‐498 targets the 3′‐UTR of the *BCL‐2* gene and inhibits Bcl‐2 protein expression. Bcl‐2 suppresses the apoptosis of colorectal cancer cells. Therefore, miR‐498 promotes colorectal cancer cell apoptosis via targeting Bcl‐2. The present discovery of the miR‐498–Bcl‐2 interaction identifies new clinical targets for therapeutic intervention of colorectal cancer.

**Abbreviations**
CRC: colorectal cancer
DLRA: dual‐luciferase reporter assay
miR‐498: microRNA‐498
miRNA: microRNA
MTT: 3‐(4,5‐dimethylthiazol‐2‐yl)‐2,5‐diphenyl‐tetrazolium bromide
NC: negative control
qPCR: RNA extraction and quantitative real‐time PCR
SD: standard deviation
WT: wild‐type

Colorectal cancer (CRC) is one of the most frequent malignancies and remains the major cause of carcinoma‐related deaths worldwide 1, 2, 3. Increasing reports from the World Cancer Analysis presented that CRC is the third most common malignant tumor in males and the second most common malignant tumor in females, making it a severe threat to human health 4. Featured by the high recurrence and mortality rate, CRC causes more than 600 000 deaths per year globally 4. However, the mechanism underlying CRC tumorigenesis and pathogenesis has not yet been fully documented. Hence the characterization of molecular biomarkers is of urgent significance for better CRC diagnosis and therapeutics.

The article "MicroRNA‐498 reduces the proliferation and invasion of colorectal cancer cells via targeting Bcl‐2" was retracted in 2024. Reasons: duplicated images; unreliable data; unreliable results or conclusions.

MicroRNAs, also known as miRNAs, are a group of noncoding RNAs consisting of 22–25 nucleotides, negatively regulating a variety of target mRNAs 5. In addition, they are also involved in other biological events, including cell death or carcinoma metastasis. Low microRNA‐498 (miR‐498) expression has been reported in many malignancies. It has been widely reported that miRNAs are critical to many biological events, such as cell death or metastasis in cancer. In addition to the malignant tumors, miR‐498 has been implicated in many cellular processes. miR‐498 has been shown to be involved in the regulation of various cancers, such as ovarian cancer and esophageal squamous cell cancer 6, 7. A previous study found that miR‐498 overexpression blocks Th17 cell differentiation of peripheral blood mononuclear cells by targeting signal transducer and activator of transcription 3 (STAT3) in patients with rheumatoid arthritis 8. Regarding the role of miR‐498 in CRC, a previous study has found that CRC cell lines and colorectal adenocarcinoma tissues showed reduced expression of miR‐498, whereas overexpression of miR‐498 in colon cancer cells resulted in lower cell proliferation 9. Nevertheless, more studies are required to gain a more comprehensive insight into the underlying mechanism of miR‐498 in CRC.

The BCL‐2 family of proteins is known as an important gatekeeper to the apoptotic response. This group of structurally related proteins comprises proapoptotic and antiapoptotic members. Tumor cells were dependent on Bcl‐2 to survive 10. In response to stress signals, malignant cells may express proapoptotic activators. Some cancer cells overexpress Bcl‐2, which can dampen this proapoptotic response 11 through binding and sequestering the proapoptotic activators. In this scenario, cancer cells are thought to be ‘primed’ for apoptosis, in that they may contain sufficient amounts of the proapoptotic activators, if released from Bcl‐2, to induce programmed cell death. Cancers that depend on Bcl‐2 for survival in this way are likely to be sensitive to Bcl‐2 modulation 12. High expression of antiapoptotic protein Bcl‐2 was observed in CRC 13. Loss of Bcl‐2 expression was able to impact the survival in CRC cells 14. Another study showed that miR‐148a promotes apoptosis by targeting Bcl‐2 in CRC 15.

This study focuses on the role and mechanism of miR‐498 on CRC. Tissue samples and cell lines of CRC were used to examine the expression of miR‐498. In addition, the effect of miR‐498 overexpression on the survival and proliferation of CRC cells *in vitro* and tumorigenesis *in vivo* was also determined.

The article "MicroRNA‐498 reduces the proliferation and invasion of colorectal cancer cells via targeting Bcl‐2" was retracted in 2024. Reasons: duplicated images; unreliable data; unreliable results or conclusions.

## Materials and methods

### CRC patient specimens

In this study, a total of 20 patients with a definite diagnosis of CRC were enrolled from the Beijing Shijitan Hospital Affiliated to Capital Medical University. From these patients, samples were collected from the tumor‐adjacent normal tissues, primary tumor and metastatic tissue. All protocols had been approved by the Medical Ethics Committee of Beijing Shijitan Hospital Affiliated to Capital Medical University, with written informed consent of all of the enrolled subjects. The study methodologies conformed to the standards set by the Declaration of Helsinki.

### Ethics statement

All experiments relating to the patients were conducted under the regulation of Animal Management Rule of the Chinese Ministry of Health (documentation 55, 2001), whereas animal experiments under the regulation of standard operating procedures were approved by the Committee on the Use and Care of Animals at Beijing Shijitan Hospital Affiliated to Capital Medical University.

### Cell culture

HT‐29, LOVO and HcoEpiC (normal cell) cell lines were obtained from Nanjing Cobioer Biotechnology Co. Ltd. (Nanjing, Jiangsu, China). HcoEpiC cells were cultured at 37 °C under 5% CO_2_ in Dulbecco's modified Eagle's medium, supplemented with 10% FBS. HT‐29 and LOVO cells were cultured in McCoy's 5a Modified and F‐12K medium, respectively.

### Cell transfections

miR‐498 mimic (5′‐UUU CAA GCC AGG GGG CGU UUU UC‐3′) and the corresponding negative control (NC mimic, 5′‐UCA CAA CCU CCU AGA AAG AGU AGA‐3′) were synthesized from RiboBio (Guangzhou, China), then transfected into HT‐29 and LOVO cells. The full‐length open reading frame of Bcl‐2 was amplified using the primers (F: 5′‐CGA GCT CAC GCC AGG TCA AGT TA‐3′, R: 5′‐CCG CTC GAG GGG GCT AGC CTC ATG A‐3′) and inserted into the upstream of pCDNA3.1 plasmid (V79020; Thermo Fisher, Waltham, MA, USA) by GenScript (Beijing, China). Cotransfection of miR‐498 mimic and pcDNA–Bcl‐2 was conducted using Lipofectamine 2000 Reagent.

### Immunoblotting

Whole‐cell lysate was prepared by incubating cells with the protease inhibitor cocktail (05892970001; Roche, Basel, Switzerland) and radioimmunoprecipitation assay buffer (pH 8.0). BCA (bicinchoninic acid) kit (23225; Thermo Fisher) was employed to detect the concentration of proteins. Proteins were then subjected to SDS/PAGE and transferred electrically onto the poly(vinylidene difluoride) membrane (Millipore, Burlington, NJ, USA). The unoccupied sites on the membrane were blocked by incubation with the primary antibodies overnight at 4 °C, followed by washing in TBST. The primary antibodies included anti‐Bcl‐2 IgG (1 : 1000, 3498; CST, Danvers, MA, USA), anti‐Bax IgG (1 : 1000, 2774; CST) and anti‐actin IgG (1 : 5000, sc‐10731; Santa Cruz, Santa Cruz, PA, USA). Then immunoblots were detected by incubating with the secondary antibodies for 1 h at room temperature. Then, after several washes in TBST, bands on the membrane were developed by using the SuperSignal West Femto Maximum Sensitivity Substrate Kit (Thermo Fisher).

The article "MicroRNA‐498 reduces the proliferation and invasion of colorectal cancer cells via targeting Bcl‐2" was retracted in 2024. Reasons: duplicated images; unreliable data; unreliable results or conclusions.

### RNA extraction and quantitative real‐time PCR

Total RNA was isolated from the CRC cells and tissue samples (100 mg) using the TRIzol reagent (15596018; Thermo Fisher) and subjected to the concentration assessment using the NanoDrop 2000 (*A*_260_). Reverse transcription was conducted to prepare cDNA using the MMLV First‐Strand Kit (Invitrogen, Carlsbad, CA, USA) and Oligo (dT) 20 Primer. cDNA was prepared for RNA extraction and quantitative real‐time PCR (qPCR) using the SYBR Select Master Mix (Invitrogen). qPCR detections of the miR‐498 and U6 were conducted using the corresponding kits, and all operations were performed. The primer sequences were as follows: miR‐498 F: 5′‐GGT TTG AAG CCA GGC GGT TTC‐3′, miR‐498 R: 5′‐CAG TGC AGG GTC CGA GGT AT‐3′; Bcl‐2 F: 5′‐CCT GTG GAT GAC TGA GTA CC‐3′, Bcl‐2 R: 5′‐GAG ACA GCC AGG AGA AAT CA‐3′; Bax F: 5′‐GTT TCA TCC AGG ATC GAG CAG‐3′, Bax R: 5′‐CAT CTT CTT CCA GAT GGT GA‐3′; U6 F: 5′‐CTC GCT TCG GCA GCA CA‐3′, U6 R: 5′‐AAC GCT TCA CGA ATT TGC GT‐3′; GAPDH F: 5′‐TGC ATC CTG CAC CAC CAA CT‐3′, GAPDH R: 5′‐TGC CTG CTT CAC CAC CTT C‐3′. U6 or GAPDH mRNA expressions were used as the internal reference. The expressions of target mRNAs were quantified by using the $2^{-\Delta \Delta C_{T}}$ method. All tests were performed in triplicates.

### 3‐(4,5‐Dimethylthiazol‐2‐yl)‐2,5‐diphenyl‐tetrazolium bromide assay

After treatment with 3‐(4,5‐dimethylthiazol‐2‐yl)‐2,5‐diphenyl‐tetrazolium bromide (MTT) reagent (20 μL, 0.5 mg·mL^−1^, V13154; Thermo Fisher), cells were incubated with DMSO (150 μL) for 10 min. The viability of cells was measured by determining *A*_490 nm_.

### Apoptosis detection

Cell apoptosis was evaluated using flow cytometry with Annexin V–FITC/propidium iodide apoptosis detection kit (556547; BD Pharmingen, Franklin Lakes, NJ, USA). Cell suspension was prepared in 20 µL of binding buffer, followed by treatment in 10 µL of Annexin V–FITC and 5 µL of propidium iodide. The apoptotic rate of cells was measured using a flow cytometer.

### Dual‐luciferase reporter assay

To identify whether miR‐498 targets Bcl‐2, we subjected WT and mutant 3′‐UTR of the BCL‐2 to dual‐luciferase reporter assay (DLRA). The wild‐type (WT) and mutated 3′‐UTRs of the *BCL‐2* gene (position 354–361 of *BCL2* 3'‐UTR) were synthesized and cloned into the XbaI site downstream of PGL3. HEK293T cells were transfected with WT/mutated Bcl‐2 and miR‐498/NC mimic for 36 h. In light of firefly luciferase sequences, luminance was calibrated, and Renilla luciferase was used for the reference luminance by using Dual‐Luciferase® Reporter Assay System (E1910; Promega, Madison, WI, USA).

The article "MicroRNA‐498 reduces the proliferation and invasion of colorectal cancer cells via targeting Bcl‐2" was retracted in 2024. Reasons: duplicated images; unreliable data; unreliable results or conclusions.

### targetscan prediction

We used the prediction algorithm targetscan to identify targets of miR‐498. The TargetScan website (http://www.targetscan.org) lists predictions according to the prediction of targeting efficacy 16. As an alternative, predictions are also ranked by their probability of conserved targeting 17.

### *In vivo* tumorigenesis experiment

Tumor formation ability was determined in an *in vivo* experiment with BALB/c nude mice as subjects. All nude mice were subjected to the subcutaneous inoculation of HT‐29 NC and HT‐29–miR‐498 cells at a density of 2 × 10^6^ cells per 0.2 mL. Tumor size was measured every 5 days after inoculation, and 30 days later, tumors were isolated from the mice that had been executed for measurement of the volume using the equation: *A* × *B* ^2^/2 (*A* is the largest diameter; *B* is the diameter perpendicular to *A*).

### Statistical analysis

All data were expressed as means ± standard deviation (SD). Comparisons among different groups were carried out with one‐way ANOVA, and a *t*‐test was used for comparison between two groups. A *P*‐value *<*0.05 indicated a significant difference.

## Results

### miR‐498 is down‐regulated in CRC tissue samples and cell lines

qPCR analysis revealed that miR‐498 expression was down‐regulated in CRC samples compared with that in the normal control group (Fig. 1A). In HT‐29 and LOVO cell lines, miR‐498 expression was lower in comparison with that in the normal colonic epithelial cell line (Fig. 1B). Thus, CRC may suppress the expression of miR‐498.

**Figure 1:** miR‐498 expression in CRC tissue samples and cell lines. (A) miR‐498 expression in CRC tissue samples and normal tissue samples (*n* = 20 and 10, respectively) analyzed using qPCR. (B) miR‐498 expression in CRC cell lines and normal colonic epithelial cell line (HcoEpiC). *n* = 3. Data are expressed as means ± SD. *P < 0.05 indicated a statistically significant difference when compared with the normal control. Comparisons among two groups were carried out with Student's *t*‐test.

### miR‐498 mimic suppresses the proliferation and induces apoptosis of CRC cells

MTT assay revealed that with increased expression of miR‐498 (Fig. 2A,B), the proliferation of HT‐29 and LOVO cell lines significantly decreased at 24–96 h after transfection when compared with the NC groups (Fig. 2C,D).

The article "MicroRNA‐498 reduces the proliferation and invasion of colorectal cancer cells via targeting Bcl‐2" was retracted in 2024. Reasons: duplicated images; unreliable data; unreliable results or conclusions.

**Figure 2:** Effect of miR‐498 overexpression on CRC cells. (A, B) Expression of miR‐498 in HT‐29 and LOVO cells transfected with either miR‐498 mimic or NC mimic measured by qPCR. (C, D) Viability of HT‐29 and LOVO cells determined at 24, 48 and 96 h by MTT assay. *n* = 3. Data are expressed as means ± SD. *P < 0.05, **P < 0.01 indicated a statistically significant difference when compared with the normal control. Comparisons among two groups were carried out with Student's *t*‐test.

Furthermore, flow cytometers were used to illustrate the role of miR‐498 in decreasing the viability of CRC cell lines. Results showed that cells transfected by miR‐498 mimic exhibited a higher cell apoptotic rate when compared with the NC group (Fig. 3A,B). Variations in Bcl‐2 and Bax expressions were detected, and the results showed that miR‐498 mimic transfection resulted in a decrease in Bcl‐2 expression but an increase in Bax expression compared with the NC group (Fig. 3C,D).

**Figure 3:** miR‐498 mimic induced apoptosis of CRC cells. (A, B) Cell apoptosis detected by the Annexin V–FITC and propidium iodide flow cytometer. Apoptotic cells are represented in the upper right quadrant of each plot. (C, D) Overexpression of miR‐498 regulated Bcl‐2 and Bax expression in the HT‐29 and LOVO cells transfected with the miR‐498 mimic or NC mimic. PIPE‐A, Propidium Iodide phycoerythrin‐A

### **miR‐498 targets 3**′**‐UTRs of Bcl‐2**

In this study, Bcl‐2 was found to be up‐regulated in the CRC cells compared with the normal colonic epithelial cells (Fig. 4A), and further experiments also showed up‐regulation of Bcl‐2 mRNA expression (Fig. 4B). Besides, bioinformatics analysis also showed that the 3′‐UTR of Bcl‐2 may be the target of miR‐498 12, 13 (Fig. 4C). Based on these findings, we conducted DLRA to verify the correlation between them. As shown in Fig. 4D, the luciferase activity was significantly decreased after miR‐498 mimic transfection as compared with other control groups. In addition, we found that the protein expression of Bcl‐2 was reduced in cells with miR‐498 overexpression (Fig. 4E,F). Thus, miR‐498 may specifically target the 3′‐UTRs of Bcl‐2.

**Figure 4:** miR‐498 targets 3′‐UTR of Bcl‐2. (A) mRNA expression of mammalian target of rapamycin (mTOR) determined by qPCR. (B) Protein expression of mTOR determined by western blotting in the CRC cell lines. (C) Graphical representation of the conserved miR‐498 binding motif at the 3′‐UTRs of Bcl‐2. (D) The luciferase activity displayed by the luciferase reporter construct. (E, F) Protein expression of Bcl‐2, after transfection of miR‐498 mimic or NC, by western blot. *n* = 3. Data are expressed as means ± SD. *P < 0.05 indicated a statistically significant difference when compared with the normal control. Comparisons among two groups were carried out with ANOVA.

The article "MicroRNA‐498 reduces the proliferation and invasion of colorectal cancer cells via targeting Bcl‐2" was retracted in 2024. Reasons: duplicated images; unreliable data; unreliable results or conclusions.

### Bcl‐2 overexpression suppresses the expression of miR‐498 in CRC cells

The earlier findings established that miR‐498 up‐regulation could affect numerous properties of CRC cells in which the role of Bcl‐2 remains unknown. Thus, in cells transfected by the miR‐498 mimic, Bcl‐2 overexpression was induced (Fig. 5A,B). In addition, Bcl‐2 depletion enhanced the survival of CRC cells by enhancing their proliferation, as revealed by the MTT assay (Fig. 5C,D), whereas in the case of Bcl‐2 overexpression, the apoptotic rate of cells was significantly decreased (Fig. 5E,F). Thus, Bcl‐2 expression might be critical to the restoration of the miR‐498‐mediated inhibition of cell proliferation.

**Figure 5:** Bcl‐2 expression rescues CRC cells. (A, B) Protein expression of Bcl‐2 in the HT‐29 and LOVO cells transfected with different vectors. (C, D) Proliferation of HT‐29 and LOVO cells overexpressing Bcl‐2. (E, F) Apoptosis of HT‐29 and LOVO cells overexpressing Bcl‐2. *n* = 3. Data are expressed as means ± SD. PIPE‐A, Propidium Iodide phycoerythrin‐A.

### miR‐498 influences CRC development in nude mouse

After subcutaneous inoculation of adenoviral miR‐498‐transfected HT‐29 cells, the tumor volume in nude mice was measured to reflect the effect of miR‐498 on the tumor formation ability. In the tumor tissues, overexpression of miR‐498 was detected (Fig. 6A), and at the 30th day after inoculation, tumor volume was determined by extraction of the tumors from the sacrificed mice. Measurements showed that in comparison with the control group, tumor growth in mice with miR‐498 overexpression was reduced, and the mice exhibited a lower weight and volume of tumor (Fig. 6B,C).

**Figure 6:** miR‐498 expression inhibits xenograft CRC tumorigenesis. The HT‐29 cell line was treated for 24 h with the adenoviral miR‐498 mimic/NC mimic. (A) miR‐498 levels in the tumor samples of each group examined by qPCR. (B, C) Measurements of the tumor volume and weight at the 28th day after inoculation. *n* = 3. Data are expressed as means ± SD. *P < 0.05 indicated a statistically significant difference when compared with the NC group. Comparisons among two groups were carried out with Student's *t*‐test.

## Discussion

Tumorigenesis is a sophisticated, synergetic process with extensive involvement of a variety of oncogenes and tumor suppressor genes. The evidence from increasing studies is not yet sufficient to illustrate the underlying mechanisms of CRC. In this study, miR‐498 was remarkably down‐regulated in both CRC tissue samples and cell lines, and the DLRA results indicated that the 3′‐UTR of Bcl‐2 is a direct target of miR‐498. Among CRC cells overexpressing miR‐498, both cell viability and proliferation were inhibited significantly, with enhanced apoptosis. However, these effects were reversed by Bcl‐2 overexpression. Thus, miR‐498 may suppress CRC by targeting *Bcl‐2* gene.

The article "MicroRNA‐498 reduces the proliferation and invasion of colorectal cancer cells via targeting Bcl‐2" was retracted in 2024. Reasons: duplicated images; unreliable data; unreliable results or conclusions.

Bcl‐2 family proteins belong to key regulators of apoptosis, which can cause various pathological consequences, including the development of cancer 18. The antiapoptotic protein Bcl‐2 is an essential member of the Bcl‐2 family, which mediated the release of proapoptotic factors responsible for the activation of caspases by stabilizing the mitochondrial outer membrane 19. Accumulating evidence suggested that Bcl‐2 expression may be associated with prognosis in malignancies, including CRC 20. Expression of Bcl‐2 has been shown to correlate with favorable clinicopathological parameters and better prognosis 21, 22, 23. The balance between proapoptotic Bax and antiapoptotic Bcl‐2 in cells can determine the cellular fate. Previous study has shown the potential prognostic and predictive significance of Bax and Bcl‐2 gene expression and Bax/Bcl‐2 ratio in CRC, and found that Bax/Bcl‐2 ratio was statistically correlated with age and tumor location. Patients with age older than 50 years showed decreased levels of Bax/Bcl‐2 ratio. Moreover, the Bax/Bcl‐2 ratio was significantly lower in tumors resected from colon compared with sigmoid colon, rectosigmoid and rectum tumors 24. In the present study, we found that miR‐498 up‐regulation reduced the expression of Bcl‐2, whereas it induced the Bax expression, suggesting that miR‐498 up‐regulation could increase the Bax/Bcl‐2 ratio, which is associated with patient age and tumor location. Therefore, miR‐498 may serve as a potential molecular marker of CRC.

In this study, after overexpression of Bcl‐2 in CRC cells transfected with miR‐498 mimic, we found that Bcl‐2 played an oncogenic role in CRC cells, as evidenced by their restored proliferation and survival and reduced apoptosis, in contrast with the function of miR‐498. In conclusion, miR‐498 may exhibit an inhibitory effect on the tumor development and progression of CRC. Overexpression of miR‐498 decreases the growth of CRC cells. Thus, miR‐498 is a promising target for the diagnosis and treatment of CRC.

## Conflict of interest

The authors declare no conflict of interest.

## Author contributions

TW conceived and designed the project. LM and LD acquired the data. WL and HG analyzed and interpreted the data. WL wrote the paper.
